The article "Plasma Levels of Vitamin A in Early Pregnancy and Correlationship with Hypertensive Disorder" was published in 2022. Journal: Comput Math Methods Med.

# Plasma Levels of Vitamin A in Early Pregnancy and Correlationship with Hypertensive Disorder

**DOI:** 10.1155/2022/3081720

**Published:** 2022-05-18

**Authors:** Jing Lv, Yunfeng Wang, Yuhua Zhao, Yingdong He, Huixia Yang, Huijing Zhang, Xiaoyu Wang

**Affiliations:** ^1^Department of Obstetrics and Gynecology, The Capital Medical University Mi Yun Teaching Hospital, Beijing 100000, China; ^2^Department of Obstetrics and Gynecology, Peking University First Hospital, Beijing, China

## Abstract

*Objective.* Analyzing the vitamin A content in early pregnancy and finding out the relationship between the serum levels of vitamin A of pregnant women and hypertensive disorder*. Method.* A total of 4,188 pregnant women who had took part in vitamin A testing in Miyun District Hospital from November 2016 to March 2020 were collected. The serum levels of vitamin A were determined by high performance liquid chromatography, and clinical and testing data were collected for statistical analysis. The original data outcome was finally analyzed with the SPSS*. Results.* 266 Hypertensive disorder cases and 2836 normal pregnancy cases were analyzed with 27 cases of twin pregnancy, 315 cases without follow-up and 744 of diabetic pregnancies excluded. The 266 women were divided into four groups: 110 women were diagnosed gestational hypertension, 65 women were diagnosed preeclampsia, 78 women were diagnosed pregnancy with chronic hypertension, and 13 women were diagnosed chronic hypertension with preeclampsia. The results shows that vitamin A level of the hypertensive group was 0.46(±0.08) mg/L, 0.47 (±0.012) mg/L, 0.47 (±0.09) mg/L, and 0.52 (±0.012) mg/L, respectively, while the level of normal group was 0.44 (±0.09) mg/L. We found that there were differences between the normal pregnant group and the preeclampsia group with statistical significance (*P* < 0.05). The difference between the pregnancy with chronic hypertension group and the normal group was statistically significant (*P* < 0.05). The difference between the chronic hypertension with preeclampsia group and the normal group was also statistically significant (*P* < 0.05)*. Conclusion.* Serum levels of vitamin A in early pregnant women have a certain correlation with the hypertensive disorder.

## 1. Introduction

Hypertensive disorder complicating pregnancy (HDCP) is a common obstetric disease that will occur in 5%-10% of all pregnancy cases, and the resultant maternal deaths account for about 10%-16% of the total number of pregnancy-related deaths, making it the second leading cause for maternal deaths. The main symptoms include hypertension, proteinuria, and edema. The purpose is to prevent the occurrence of severe preeclampsia and eclampsia, reduce the perinatal morbidity and mortality of the mother and the baby, and improve the prognosis of the mother and the baby. Preeclampsia may affect multiple organs and systems of the mother, cause hypoxia, restrict growth and development of the baby, and endanger the life safety of the mother and the baby [1]. The incidence of preeclampsia in the world is about 2%-5%, and the incidence in our country is about 9.4%, so it is a medical difficulty recognized by the global public health undertaking [2]. For preeclampsia, most scholars emphasize early monitoring and intervention. In recent years, studies have found that in addition to genetic, metabolic and immunological factors, oxidative stress injury also plays an important role in the pathogenesis of preeclampsia [3]. The patients with preeclampsia will experience placental ischemia and hypoxia, which are manifested by increase in pro-oxidant substances and decrease in antioxidant substances, so recognizing the unbalance of the oxidation and antioxidant systems of pregnant women may be helpful for the early diagnosis of preeclampsia. Based on the above theories, the studies on supplementing antioxidants to prevent preeclampsia are also increasing gradually. Some studies have shown that antioxidants can effectively reduce the oxidative stress response, thus reducing the incidence of preeclampsia in pregnant women and improving the adverse outcomes of pregnant women and perinatal infants [4].

As more and more studies correlate the levels of vitamin A strong antioxidants in the body to the development of preeclampsia during pregnancy, the correlation between the serum levels of pregnant women in early pregnancy and pathogenesis of the HDCP is rarely reported at home and abroad. This study is a large-sample clinical study that adopts retrospective analysis to explore the correlation between serum levels of vitamin A in pregnant women at 12 weeks of pregnancy and the HDCP and discuss whether they can be used as clinical testing indicators.

## 2. Data and Methods

A sample a total of 4,188 pregnant women who had undergone routine obstetric examination (preliminary screening) in our hospital from November 2016 to May 2020 were selected. They all signed the informed consent form, and their blood samples and clinical information were collected. Then, 27 cases of twin pregnancy and 315 cases without follow-up were excluded. Finally, a total of 3846 cases were analyzed. Among them, after excluding 744 cases of DM and GDM cases, our study had 266 cases with HDCP, which was the case group, and 2836 cases in the control group.

### 2.1. Criteria

#### 2.1.1. Diagnostic Criteria of Case Group

Refer to *Obstetrics and Gynecology* (9th Edition) compiled by Xie Xing; the specific diagnostic criteria are as follows:

1. Gestational hypertension: Hypertension occurs after 20 weeks of pregnancy, systolic blood pressure ≥140 mmHg, and (or) diastolic blood pressure ≤90 mmHg, which return to normal levels within 12 weeks after delivery; urine protein (-)
2. Preeclampsia: the blood pressure ≥140/90 mmHg after 20 weeks of pregnancy; urine protein ≥0.3 g/24 h or random urine protein (+), which may be accompanied by upper abdominal discomfort, headache, and other symptoms. Severe preeclampsia includes Preeclampsiaand also the following: (1) systolic blood pressure ≥160-180 mmHg or diastolic blood pressure ≥110 mmHg; (2) 24 h urine protein >2.0 g or random urine protein (+++) or above; (3) central nervous system dysfunction, mental status change, severe headache (frequent, not relieved by conventional analgesics), cerebrovascular accident, blurred vision, punctate hemorrhage in the fundus, and very few patients that may suffer cortical blindness; (4) hepatocyte dysfunction, hepatocellular injury, and serum transaminase that is at least 2 times higher; (5) upper abdomen or upper right quadrant pain and other symptoms of liver capsule swelling, subcapsular hemorrhage of the liver, or hepatic rupture; (6) oliguria, 24 h urine volume <500 mL; (7) pulmonary edema and heart failure; (8) platelets <100 × 10^9^/L and coagulation disorders; (9) microangiopathic hemolysis and elevated blood lactate dehydrogenase; and (10) fetal growth restriction, oligohydramnios, and placental abruption
3. Pregnancy with chronic hypertension: systolic blood pressure ≥140 mmHg before 20 weeks of pregnancy and/or diastolic blood pressure ≤90 mmHg (excluding trophoblastic diseases), which do not aggravate significantly during pregnancy, or the hypertension first diagnosed after 20 weeks of pregnancy continues until 12 weeks after delivery
4. Chronic hypertension with preeclampsia: Chronic hypertension without urine protein before pregnancy, but proteinuria occurs after 20 weeks of pregnancy; or proteinuria exists before pregnancy and increases significantly after pregnancy; or blood pressure further increases, or thrombocytopenia occurs (<100 × 10^9^/L), or other serious manifestations occur, such as liver and kidney damages, pulmonary edema, neurological abnormalities, or visual disturbances

### 2.2. The Control Group Consists of Healthy Pregnant Women with Single L4ive Births and without any Pregnancy Complication

#### 2.2.1. Testing Method

3-5 ml of fasting peripheral venous blood of the research object was collected, while anticoagulant treatment is not needed. After high-speed centrifugation of the blood, the upper serum was sucked with a pipette and was stored at a low temperature of -20°C away from light. The content of vitamin A in serum was determined by high performance liquid chromatography, and the standard curve was drawn according to the sample concentration on high performance liquid chromatograph. An automatic biochemical analyzer was used to test contents of vitamin A. The test results of this study were provided by Beijing Harmony Health Medical Laboratory. The mass concentrations of vitamin A in pregnant women's serum were determined by high performance liquid chromatography (model: Agilent UPLC1290), and the test instrument was provided by Agilent Technologies Co. Ltd. Before blood drawing, pregnant women should be asked to go on an empty stomach for more than 8 hours, and about 4 ml of peripheral venous blood needs to be collected, while anticoagulant treatment is not needed. The blood should be stored and transported at 0-4°C away from light. After obtaining blood samples, they should be centrifuged in time to obtain serum. Serum samples need to have deproteinization and impurities treatment, and then n-hexane is added to extract effective components. The upper serum is taken, dried, and then redissolved with methanol. The effective components of it are tested, and the mass concentrations of vitamins A and E are measured. The standard curve equation of serum samples was made by the deproteinization data and standard substance data tested with instruments, and the relative standard deviation was less than 15%, x±2 s.

#### 2.2.2. Reference Standards

Normal body reference value: Serum vitamin A level is of 0.3-0.7 mg/L, respectively. If the value is lower than the lower limit of reference value, it will be regarded as inadequate for the body; if the value is higher than the upper limit of reference value, it will be regarded as excessive for the body.

### 2.3. Statistical Method

All collected complete data were entered into Excel successively, and SPSS 23.0 software was used for statistical analysis. Serum vitamin A were expressed as mean ± standard deviation (x ± s), and test was used for comparison between the two groups. *P* < 0.05 is considered statistically significant. All count data are expressed as percentages (%), and the test method adopts the X^2^ test statistical method; *α* = 0.05 is the reference standard, and *P* < 0.05 means that the difference is statistically significant.

## 3. Results

The range of vitamin A is 0.2-1.2 mg/L. Finally, data from 266 cases of hypertensive disorders was collected and analyzed, along with 2836 cases of the normal pregnancy. The demographic details are shown in Table 1.

### 3.1. Comparison of Vitamin A Concentration between the Case Group and the Control Group

The serum vitamin A level was 0.47 (±0.099) mg/L for the case group and 0.44 (±0.091) mg/L for the control group; the comparison between the two groups showed *P* < 0.001, so the difference was statistically significant (*P* < 0.05) (see Table 2).

### 3.2. Comparison of Vitamin A Concentrations between the Subgroups of the Case Group and the Control Group

The subgroups of the case group contained 110 cases of hypertensive disorder complicating pregnancy, 65 cases of preeclampsia, 78 cases of pregnancy with chronic hypertension, and 13 cases of chronic hypertension with preeclampsia. The level of vitamin A in the hypertensive disorder complicating pregnancy subgroups was higher than that of the control group. The difference between the preeclampsia group and the control group, between chronic hypertension group and the control group, and between chronic hypertension with preeclampsia group and the control group were all statistically significant (*P* < 0.05). However, the difference of vitamin A between gestational hypertension group and control group was not statistically significant (*P* > 0.05). See Table 3.

## 4. Discussion

At present, the global maternal mortality caused by hypertensive disorder complicating pregnancy is as high as 14% [5]. Current studies conclude that oxidative stress injury is the main pathogenesis [6]. The oxidative damage process caused by the large accumulation of reactive oxygen species (ROS) free radicals in the body promotes an inflammatory response [7]. Therefore, many studies have shown that oxidative stress is a central link in the pathogenetic process of preeclampsia [8]. Vitamin A belongs to the non-enzymatic strong antioxidants in the antioxidant defense system of human body and has the functions of anti-oxidation, scavenging free radicals, and anti-apoptosis; if vitamin A has excess or deficiency, it will cause physical abnormalities [9]. Related studies show that vitamin A can maintain the integrity of the epithelial tissue structure, have antioxidation effect, and affect the immune and reproductive system functions of organism [10] and can reduce damage of organism through a variety of ways [11]. If that content in pregnant women is low, it will cause the accumulation of excessive free radicals, which will cause damage to the placental vascular endothelium and increase the risk of adverse pregnancy outcomes [12]. When pregnant women suffer hypertensive disorders complicating pregnancy, vitamin A also changes accordingly. Therefore, the detection of serum levels of vitamin A can be used as a means to monitor preeclampsia.

At present, most of the study results obtained based on the third trimester of pregnancy and after the fetal delivery show that the oxidative stress markers (e.g., malondialdehyde) in the serum and placenta of pregnant women with preeclampsia increase significantly, while the levels of antioxidant markers (e.g., vitamin C and vitamin E) decrease significantly [13–16]. At present, the studies on the correlation between vitamin A and the hypertensive disorder complicating pregnancy (HDCP) are very controversial [17]. As more and more studies are focusing on oxidative stress response in the pathogenesis of HDCP, the studies on strong antioxidant vitamins are also increasing.

In our study, the serum levels of vitamin A in the gestational hypertension group were close to those in the control group, while the values of the preeclampsia group, the pregnancy with chronic hypertension group, and the chronic hypertension preeclampsia group were higher than those of the control group. When comparing the vitamin A levels of the preeclampsia group with the control group, the difference was statistically significant. The related study results of Zhao et al. showed that the serum vitamin A level of PE pregnant women at 12-20 weeks of pregnancy was higher than that of healthy control group, which showed the seminal result as ours [18]. However, in the study of Li et al., the serum levels of vitamin A of patients in the preeclampsia group were lower than those of the pregnant women in healthy control group, especially the serum levels of vitamin A in patients with severe preeclampsia, which were significantly lower than those in patients with mild preeclampsia [19]. Therefore, the studies on the levels of antioxidant vitamins have not reached a unified conclusion.

The reasons leading to these inconsistent conclusions contained the following: (1) This study only obtains the serum vitamin levels at 12 weeks of pregnancy, and does not record the serum vitamin A levels of pregnant women after 12 weeks of pregnancy. In consideration that the serum levels change significantly from the first trimester to the third trimester, the serum levels in the third trimester cannot be recorded for statistical comparison, so the specific conclusions need to be further studied, and the serum levels in the second and third trimesters need to be tested for comparison and analysis [20]. (2) The serum vitamin A may have a certain correlation with different diets of pregnant women in the first trimester, especially the regional differences and the enhancement of health care awareness in early pregnancy, the intake of multiple multivitamins, and the level of progesterone in the body, leading to changes in serum vitamin levels [21]. (3) The number of cases of preeclampsia and chronic hypertension with preeclampsia is small, which is because our hospital is a district-level hospital, some of the cases lost to follow-up are critically ill pregnant and lying-in women who need to be referred to a higher-level hospital, and the follow-up results are not tracked, resulting in low acquisition rate of preeclampsia incidence; a large number of data and prospective studies are still needed for further support.

To sum up, as a critical disease in obstetrics, the hypertensive disorder complicating pregnancy attacks insidiously and rapidly and has a serious impact on the mother and the baby. Early identification, early management, and early intervention can significantly reduce the adverse outcomes of pregnant women and perinatal infants. Vitamins are strong antioxidants in the body. In this study, vitamin A is related to the onset of the hypertensive disorder. However, regardless of the gestational weeks when vitamin A is obtained or the prevention and explanation of the development and progression processes of preeclampsia through external supplementation of vitamins, we need to further strengthen and improve the follow-up, increase the sample size of the case group, improve the monitoring values of vitamin A during the second and third trimesters, and analyze and improve the conclusions for clinical guidance.

## Figures and Tables

**Table 1:** Demographic data.

Item	Mean (SD)/*n* (%)
Age	30.05 (4.33)
<35 years old	3192 (83)
≥35 years old	654 (17)
Obesity (BMI ≥25)	191 (5)
DM	88 (2.3)
GDM	656 (80.7)
Hypertensive disorder	
Gestational hypertension	140 (3.6)
Preeclampsia	83 (2.2)
Pregnancy with chronic hypertension	112 (2.9)
Chronic hypertension with preeclampsia	16 (0.4)
Outcome	
Gestational age at delivery	37.6 (1.31)
Preterm birth (<37 gestational weeks)	807 (21)
Birth weight	3364.97 (546.32)

**Table 2:** Comparison of vitamin A concentration between the case group and the control group.

Group	Number of cases	Vitamin A
Case group	266	0.47 (±0.099)
Control group	2836	0.44 (±0.091)
*t* Value		-4.505
*P* value		<0.001

**Table 3:** Comparison of vitamin A concentrations between the subgroups of the case group and the control group.

Group	N (%)	Mean	*P* value
Hypertensive disorder			
Gestational hypertension	110 (3.5)	0.46 (0.08)	0.055
Preeclampsia	65 (2.1)	0.47 (0.12)	0.01
Pregnancy with chronic hypertension	78 (2.5)	0.47 (0.09)	0.006
Chronic hypertension with preeclampsia	13 (0.4)	0.52 (0.12)	0.002
Control	2836 (91.4)	0.44 (0.09)	

## Data Availability

The data used to support the findings of this study are available from the corresponding author upon request.

## References

[1] Capriglione S., Plotti F., Terranova C. (2020). Preeclampsia and the challenge of early prediction: reality or uto-pia? State of art and critical review of literature. *The Journal of Maternal-Fetal & Neonatal Medicine*.

[2] Li X., Tan H. Z., Huang X. (2016). Similarities and differences between the risk factors for gestational hypertension and preeclampsia: a population based cohort study in South China. *Pregnancy Hypertens*.

[3] Weissgerber T. L., Gandley R. E., McGee P. L. (2013). Haptoglobin phenotype, preeclampsia risk and the efficacy of vitamin C and E supplementation to prevent preeclampsia in a racially diverse population. *PLoS One*.

[4] Talaulikar V., Manyonda I. (2010). The myth of vitamins C and E for the prevention of preeclampsia: Just when will the penny drop. *American Journal of Obstetrics and Gynecology*.

[5] Smith T. A., Kirkpatrick D. R., Kovilam O., Agrawal D. K. (2015). Immunomodulatory role of vitamin D in the pathogenesis of preeclampsia. *Expert Review of Clinical Immunology*.

[6] Redman C. W., Sargent I. L. (2000). Placental debris, oxidative stress and pre-eclampsia. *Placenta*.

[7] Guan Z., Li H. F. (2014). The relationship between oxidative stress effect and gestational hypertension disease. *Chinese Journal of Clinical Physicians (Electronic)*.

[8] Burton G. J., Jauniaux E. (2011). Oxidative stress. *Best Pract Res Clin ObstetGynaecol*.

[9] Omur A., Kirbas A., Aksu E. (2016). Effects of antioxidant vi- tamins (A, D, E) and trace elements (Cu, Mn, Se, Zn) on some metabolic and reproductive profiles in dairy cows during transition period. *Polish Journal of Veterinary Sciences*.

[10] Patel S., Akalkotkar A., Bivona J. J. (2016). Vitamin A or E and a catechin synergize as vaccine adjuvant to enhance im- mune responses in mice by induction of early interleukin-15 but not interleukin-1 responses. *Immunology*.

[11] Weissgerber T. L., Gandley R. E., McGee P. L. (2015). Influence of vitamin C and vitamin E on redox signaling: implications for exercise adaptations. *Free Radical Biology & Medicine*.

[12] Rumbold A., Ota E., Hori H., Miyazaki C., Crowther C. A. (2015). Vitamin E supplemen- tation in pregnancy. *Cochrane Database of Systematic Reviews*.

[13] Cohen J. M., Beddaoui M., Kramer M. S., Platt R. W., Basso O., Kahn S. R. (2015). Maternal antioxidant levels in pregnancy and risk of preeclampsia and small for gestational age birth: a systematic review and meta-analysis. *PLoS One*.

[14] Oostenbrug G. S., Mensink R. P., Al M. D., van Houwelingen A. C., Hornstra G. (1998). Maternal and neonatal plasma antioxidant levels in normal pregnancy, and the relationship with fatty acid unsaturation. *The British Journal of Nutrition*.

[15] Calfee-Mason K. G., Spear B. T., Glauert H. P. (2004). Effects of vitamin E on the NF-kappa B pathway in rats treated with the peroxisome proliferator, ciprofibrate. *Toxicology and Applied Pharmacology*.

[16] Das B., Saha-Roy S., Das Gupta A., Lahiri T. K., Das H. N. (2012). Assessment of placental oxidative stress in pre-eclampsia. *J ObstetGynaecol India*.

[17] Can M., Guven B., Bektas S., Arikan I. (2014). Oxidative stress and apoptosis in preeclampsia. *Tissue & Cell*.

[18] Zhao Z. Y. (2018). Pregnant women with preeclampsia serum levels of vitamin A, E correlation research.

[19] Huang L. Z. J., Zeng D D L. S., Li Z., Huang L., Zeng D. (2018). Pregnant women vitamin A and E level and the correlation of preeclampsia. *Journal of Practical Medical Journal*.

[20] Jiang H., Chen H., Ni J. J. (2015). Beijing pregnant women under routine care status quo of the serum levels of vitamin A, E. *Journal of the People's Liberation Army Medical Journal*.

[21] Cardoso P. M., Surve S. (2016). The effect of vitamin E and vitamin C on the prevention of preeclampsia and newborn outcome: a case-control study. *J ObstetGynaecol India*.

